# The Beliefs of Third-Level Healthcare Students towards Low-Back Pain

**DOI:** 10.1155/2014/675915

**Published:** 2014-04-10

**Authors:** Norelee Kennedy, John Healy, Kieran O'Sullivan

**Affiliations:** Department of Clinical Therapies, University of Limerick, Limerick, Ireland

## Abstract

*Objectives*. Beliefs held by healthcare providers are part of the complex recovery of a patient with low-back pain (LBP). The aim of this study was to investigate the attitudes and beliefs of Irish university healthcare students towards LBP. *Methods*. Physiotherapy (*n* = 107), medicine (*n* = 63), nursing, and midwifery (*n* = 101) students completed the survey. Demographic data, LBP related beliefs [Back Beliefs Questionnaire (BBQ) and the Fear Avoidance Beliefs Questionnaire physical subsection (FABQ-PA)] were collected. *Results*. Two hundred and seventy-one students responded (response rate 29%). Student physiotherapists had significantly lower FABQ (*P* < 0.001) scores than medical (95% CI [−5.492, −1.406]) and nursing students (95% CI [−7.718, −22.307]). Physiotherapy students had significantly higher BBQ scores (*P* < 0.0001) than medical (95% CI [1.490, 5.406]) and nursing students (95% CI [6.098, 11.283]). Beliefs of physiotherapy and medical students were significantly better among fourth-year year than first-year students (*P* < 0.0001) but were not significantly different for nursing students (*P* = 0.820 for FABQ and *P* = 0.810 for BBQ). *Conclusions*. Physiotherapy students had more positive beliefs towards LBP than medical and nursing students. Physiotherapy and medical students' beliefs towards LBP significantly improved over the course of their studies.

## 1. Introduction

Low-back pain (LBP) is a common problem in western countries, with some studies reporting between 83% and 91% lifetime prevalence amongst general populations [1, 2]. It has become clear that LBP is best understood from a biopsychosocial viewpoint [3, 4], which recognizes the important interactions between biological, psychological, and social aspects of a person's experience of pain [5, 6]. When considering the cognitive and psychosocial factors that are associated with LBP, fears of harm secondary to physical activity, self-efficacy beliefs, culture, gender, and fear of further injury are among the most important factors to consider [7–9]. These factors may in turn influence the beliefs a person has towards LBP, possibly contributing to potential disability [9, 10].

Beliefs held by health care providers are part of the complex recovery of a patient who has LBP [3]. Health care providers' advice, education, and recommendations may have direct influence on the recovery of a patient [3, 11, 12], and this advice may have a telling influence on the beliefs and attitudes of the patients themselves [13]. Given the influence that healthcare practitioners have on a patient's recovery, there has been relatively little study on the attitudes and beliefs held by student healthcare professionals towards LBP. There has been some investigation into this area which has looked at student nurses and physiotherapists separately [7, 12, 14, 15]. Surprisingly, there is only one which compares student nurses and physiotherapists [16], where it was found that beliefs about the inevitable consequences of LBP and fear-avoidance behaviors were more negative in student nurses when compared with student physiotherapists. Only one study [17] has compared chiropractic, medical, occupation therapy, pharmacy, and physiotherapy students and found cross-discipline differences between groups. In that study physiotherapy and chiropractic students had more positive beliefs towards LBP, and LBP beliefs influenced their recommendations on LBP vignettes.

Before commencement of full time employment, LBP is common in both student nurses and physiotherapists. Lifetime prevalence data on both of these undergraduate professions varies, with between 32% and 79% of undergraduate nurses having experienced LBP before graduation [14, 16, 18]. Studies have shown lifetime prevalence of LBP amongst student physiotherapists to be between 19% and 65% [7, 15, 16]. There is currently a lack of prevalence rates for LBP among medical students. Similarly, it is still unclear from the literature whether current or previous LBP among student physiotherapists, nurses, and doctors has an influence on attitudes and beliefs about back pain. Urquhart et al. [2] looked at attitudes and beliefs of community dwelling women towards LBP and found that while most had positive views about LBP, those who had high pain intensity at the time of testing were more pessimistic in their views. It may be interesting to find out if this pertains to student health care professionals also. Mitchell et al. [14] found that there were no significant differences in beliefs and attitudes between undergraduate nurses who did, or did not, have current LBP. Similarly, other studies [7, 15] found there were no significant differences in beliefs and attitudes between those with and without a history of LBP. Furthermore, it is unclear if students who have experienced LBP have differing attitudes to those who currently have LBP or who have never had LBP at all. Additionally, the effect of gender on LBP beliefs is unclear. Ryan et al. [15] found no significant difference between genders in attitudes towards LBP. However, it has been reported that female healthcare professionals considered pain behaviors more acceptable than their male counterparts [19]. Similarly, it has also been reported that women who have chronic musculoskeletal pain have greater pain-related disability than do men [20]. This may be pertinent to physiotherapy and nursing cohorts, where high levels of occupational LBP [18, 21] and predominance of the female gender are present. Thus, the aim of this study was to compare the beliefs of student nurses, physiotherapists, and doctors towards LBP and to investigate whether related demographic factors (current or previous LBP, gender, and year of study) have an influence on these beliefs.

## 2. Materials and Methods

### 2.1. Study Design

A cross-sectional survey was undertaken in 2012 in one university in Ireland. Students across all years in the undergraduate courses of physiotherapy (four-year program) and nursing and midwifery (four-year program) and the graduate Entry Medicine degree (four-year program) were invited to participate. Approval to undertake the study was granted by the university's Research Ethics Committee.

### 2.2. Procedure

Program directors for the three programs were contacted by the study authors and informed about the study and asked to indicate the preferred method of response to the survey (written or online survey). The survey was undertaken in the last four weeks in the final semester of the academic year. The physiotherapy students completed the survey at the end of an agreed class time. This agreed time was decided upon consultation with the physiotherapy program director and relevant lecturers. One of the authors (John Healy) met with the student groups and informed them about the survey and collected the completed surveys. The other two cohorts (medicine and nursing) were sent an electronic survey (surveymonkey.com). This email contained a hyperlink to the survey allowing students to participate. Two followup emails were sent as reminders to complete the survey. A draw for a single €100 retail voucher was offered as an incentive to all those who completed the survey.

### 2.3. Outcome Measures

The survey was designed using the Back Beliefs Questionnaire (BBQ) and the physical subsection of the Fear-Avoidance Beliefs questionnaire (FABQ-PA) as the primary measures. Other questions determined age, gender, current LBP, previous LBP, and year of study. The BBQ was developed [22] to investigate a person's beliefs about the inevitable consequences of LBP. It consists of fourteen statements aimed to examine individual's beliefs about LBP regardless of whether LBP has been previously experienced. Nine (1, 2, 3, 6, 8, 10, 12, 13, 14) of the fourteen questions are part of the questionnaire with the other five questions acting as distractors. The scale is calculated by reversing and summing the nine scores. The total score ranges from 9 to 45, with a higher score indicating more positive beliefs about LBP and lower scores indicating more negative beliefs. The measure has excellent internal consistency with a Cronbach's Alpha of 0.7 and an ICC of 0.87 [22].

The Fear-Avoidance Beliefs Questionnaire (FABQ-PA) [23] consists of two subscales for physical activity (FABQ-PA) and for work. For the purpose of this study, the FABQ-PA was used to attain a snapshot as to the level of fear-avoidant behaviors that student healthcare professionals display towards physical activity in their day-to-day lives. Four individual items are scored on a Likert scale of 0–6. Consequently, the total score ranges from 0 to 24, with a lower score indicating more positive beliefs about physical activity and a higher score more fear-avoidant beliefs towards physical activity [23]. It was shown to have good reliability and construct validity [23], where Cronbach's Alpha was reported to be 0.77 showing excellent internal consistency.

### 2.4. Data Analysis

Data was assessed for normality using a Kolmogorov-Smirnoff test and was normally distributed. Descriptive statistics were used to display the means and standard deviations for the data. Multivariate analysis of variance was used to examine overall differences in the two beliefs subscales between the three different courses. Beliefs (FABQ and BBQ) were the dependent variables with age, gender, year of study, current LBP, and previous LBP entered as covariates. The results from the Willks Lambda test were used for interpretation of the multivariate tests. Independent *t*-tests were used to further explore the significant differences identified in the multivariate tests. Data analysis was carried out using Statistical Program for the Social Sciences (SPSS) version 20.0 (SPSS Inc, Chicago, IL).

## 3. Results

A total of 271 (sixty-four males and two hundred and seven females) responded to the survey, representing an overall response rate of 29%. The mean age for the group was 22.8 years (standard deviation 4.95 years) with a range from 17 to 50 years. Demographic information and characteristics per discipline are shown in Table 1.

### 3.1. Between Group Differences

There were significant differences across the three student groups for both the BBQ (*P* < 0.001) and FABQ-PA (*P* < 0.001). Student physiotherapists had significantly higher BBQ (*P* < 0.001) and significantly lower FABQ-PA (*P* < 0.001) scores than both the medical students and nursing students. Furthermore, medical students had significantly higher BBQ scores (*P* < 0.001) than nursing students, while their FABQ-PA scores did not differ significantly (*P* = 0.225). Male students scored significantly higher on the BBQ (*P* = 0.017) with no significant differences observed for FABQ-PA scores between genders (*P* = 0.995).

Multivariate testing showed significant differences for both FABQ (*P* < 0.001) and BBQ scores (*P* = 0.002) for year of study. Further testing of individual disciplines comparing year 1 and year 4 scores indicated that there were significant differences in beliefs on both the BBQ and FABQ for physiotherapy and medical students. There was a small nonsignificant difference in nursing scores on both the FABQ and BBQ.

### 3.2. Effect of LBP Experience on Beliefs

Students currently experiencing LBP reported no difference in FABQ scores (*P* = 0.269) or BBQ scores (*P* = 0.422) from those not experiencing LBP currently. Students who have had previous LBP had significantly poorer FABQ scores (0.05) than those who have not, but there were no differences in BBQ scores (*P* = 0.393).

## 4. Discussion

This is the first study to compare beliefs towards LBP among different disciplinary year groups of healthcare students. The results of this study indicate that student physiotherapists had more positive beliefs about the inevitable consequences of LBP, as well as displaying less fear-avoidant tendencies about physical activity in their day-to-day lives when compared to their medical and nursing counterparts. A recent study [17] also reported highest mean BBQ scores for physiotherapy students, as in our study. Similar results were found in a study which reported that nursing student had significantly more negative back pain beliefs than physiotherapy students [16]. These differing attitudes and beliefs may be rooted in a number of factors, including level of pain knowledge. Interestingly, another study found the level of pain knowledge amongst final year nursing students to be generally low, which perhaps helps to explain the more negative beliefs surrounding LBP in this population [24]. Equally, a different study found that final year physiotherapy students had a greater knowledge of chronic pain mechanisms when compared to final year medical students [25]. Contrasting levels of pain knowledge amongst undergraduate healthcare practitioners may provide hypotheses as to how differing attitudes towards pain, and more specifically LBP, are shaped in this population.

Another finding of the present study was that the medical students had more positive beliefs and attitudes about the inevitable consequences of LBP than the nursing cohort, but fear-avoidant attitudes remained similar between both cohorts. The more negative fear-avoidant beliefs displayed among medical students in this study are supported by another study which showed similar results; one in six GPs was likely to provide advice against physical activity for the treatment of LBP [11]. Furthermore, it has been found that qualified physiotherapists had a greater belief that treatment could still be successful, even for those patients who were still in pain, when compared against doctors [26].

Females in the present study appeared to present with more negative beliefs and attitudes about the inevitable consequences of LBP, when compared with their male counterparts. This is in contrast to findings of a different study [15], where gender did not have an apparent effect on beliefs and attitudes towards chronic LBP in both healthcare and nonhealthcare student populations. However, there is a wealth of research conducted on gender and its effect on pain perception [19, 20, 27]. It has been found previously that male healthcare professionals have a stronger belief that treatment could be successful even if pain persisted in comparison to their female counterparts [26]. That study also noted a significant difference between male and female doctors, with female doctors having stronger beliefs that heavy or monotonous work should be avoided by patients experiencing LBP. Female health care professionals considered pain behaviors more acceptable than their male counterparts [19]. Thus these findings may provide some insight into why future female healthcare practitioners in the current study presented with poorer beliefs and attitudes in relation to the inevitable consequences of LBP. In contrast to this, the other side of the argument must be taken into consideration when reviewing the literature. In a study of back beliefs and attitudes among the general population it was found that subjects who took time off work had significantly lower BBQ scores and were more likely to be male [1].

### 4.1. Influence of LBP Experience on Beliefs towards LBP

This study found that students currently experiencing LBP did not have different BBQ or FABQ scores. However, those who had previously experienced LBP had lower FABQ scores than students who had no previous LBP. Interestingly, there was no difference on BBQ scores indicating that while those with previous LBP may display more fear-avoidant behaviors than those with no previous LBP they do not hold different beliefs on the long term consequences of that LBP. To date, the evidence on the influence LBP status can have on the beliefs and attitudes towards LBP and physical activity has been conflicting. Other studies have reported no difference in fear-avoidant beliefs between groups of students (1, 2). One study also found that those who had LBP in the past week had more negative beliefs than those who had LBP in the past but not at present, which perhaps indicates that pain intensity may have a significant effect on beliefs and attitudes towards LBP [1]. Community dwelling women who reported a high level of pain intensity and disability at the time of testing held more pessimistic views towards the inevitable consequences of LBP [2]. Previous or current experience of LBP had no impact on the beliefs and attitudes towards LBP in either Brazilian or Australian student physiotherapists [7, 13]. Furthermore, the fear-avoidant beliefs of GP's were not related to personal LBP experience [11]. However, it has also been reported in a different study that beliefs and attitudes were more negative in students without a history of LBP [16], indicating that those who had LBP previously had more positive beliefs in comparison to those who have never experienced LBP.

### 4.2. Influence of Year of Study on Beliefs towards LBP

A significant difference from first year to fourth year in beliefs surrounding the inevitable consequences of LBP and fear avoidant behaviors in relation to physical activity amongst physiotherapy and medical cohorts, but not among nursing students, was noted in this study. Differences in the beliefs of physiotherapy students towards LBP in different program years have been reported elsewhere with fourth-year physiotherapy students having more positive attitudes towards functioning in individuals with LBP than first-year physiotherapy students [15].

### 4.3. Implications for Future Research

In light of the more negative beliefs observed in nursing students, exploring the reasons for this is important. Nurses are key members of the healthcare team and their beliefs towards LBP are importantconsidering the influence a clinician has on a patient's own beliefs and attitudes [3, 11] and the high prevalence of LBP among nursing students, who had the highest percentage of current LBP among the three groups. Various methods have been used in the past to help improve beliefs and attitudes of the general population as well as student healthcare professionals. These methods include media campaigns on back pain [1, 28] teaching modules [13] and information booklets [29]. While it has been previously found that a module devoted to LBP helps the attitudes and beliefs of physiotherapy students [13], it may be an area of interest in future to investigate whether this would also pertain to those from other student healthcare degrees, particularly nursing. Not only might this improve the perceptions of LBP of among nursing students, but also, in turn, be of benefit to patients that may manage, whilst as a student but also in the future as qualified clinicians.

### 4.4. Limitations

There were some limitations found in the present study. The low response rates of both student nurses and doctors raise concerns about possible response bias. This possibility exists because the nonresponding students may have differing attitudes and beliefs from the population surveyed. However, every opportunity was given to potential participants to take part with succinct questionnaire style, monetary incentives, and followups, all of which have been shown to increase response rates among clinicians [30]. Generalisability of results is also a limitation of this study. The medical students surveyed are at graduate entry level, so therefore may have already undergone a healthcare course. This question was included in the questionnaire, but due to low response rates among the medical students, and in turn the small percentage that answered yes (*n* = 10) to this question, it was deemed unnecessary to further analyze this question. Furthermore, with the mean age being higher in medical students, they had increased opportunity over their lifetime to be exposed to LBP, than their nursing and physiotherapy counterparts. Only one university in one country is represented in this study, limiting generalizability. Confounding factors such as curricula and level of pain knowledge were not accounted for, and factors which can in turn shape the beliefs and attitudes an individual may hold about LBP [13].

## 5. Conclusion

Results from this study show that differences exist in the beliefs of three cohorts of students toward LBP. Physiotherapy students had the most positive LBP beliefs while nursing students had the most negative. Medical and physiotherapy students LBP beliefs improved significantly over their four-year degree programs, while nursing students essentially remained the same. Student with previous LBP were found to have significantly poorer levels of fear-avoidant behaviors towards LBP compared to students with no previous LBP. These findings highlight the need for education for nurses to promote positive beliefs towards LBP. Further research is required to provide evidence based recommendations of how to address these contrasting beliefs.

## Figures and Tables

**Table 1:** Profile of participants.

	Physiotherapy	Medicine	Nursing
Age (mean (SD))	21.3 (4.1)	25.9 (2.8)	22.5 (6.0)
LBP currently (%)	14.8	36.6	33.3
Gender (m/f)	34/73	22/42	9/92
Year of Study			
Year 1	31	24	20
Year 2	26	11	34
Year 3	27	17	22
Year 4	23	12	25
Past LBP (%)	73%	79%	74%
FABQ total (mean (SD))	9.18 (6.58)	11.19 (5.26)	12.52 (5.81)
BBQ total (mean (SD))	33.71 (6.31)	31.08 (5.63)	26.56 (5.41)
